# Situation of Pediatric Patients with Testicular Torsion in Times of COVID-19

**DOI:** 10.1155/2023/9960452

**Published:** 2023-05-08

**Authors:** Marta Komarowska, Małgorzata Kowalska, Kamil Grubczak, Alicja Pawelczyk, Adam Hermanowicz, Wojciech Debek, Ewa Matuszczak

**Affiliations:** ^1^Department of Pediatric Surgery and Urology, Medical University of Bialystok, Bialystok, Poland; ^2^Department of Regenerative Medicine and Immune Regulation, Medical University of Bialystok, Bialystok, Poland

## Abstract

Purpose. To assess whether the COVID-19 pandemic had an influence on presentation of testicular torsion and/or increase in the frequency of orchiectomy. *Patients and Methods.* This retrospective study included boys under 18 years of age with testicular torsion divided in two groups: pre-COVID operated in 2019 vs. COVID-19 group from 2020. We compared demographic data as well as local and general symptoms. We analyzed additional tests, intraoperative findings, length of operation and hospitalization, and followup. *Results.* We analyzed the data collected from 44 patients (24 boys from first group vs. 20 boys from second group). The median age was 13.4 years vs. 14.5 years in the latter. The median time of symptoms duration was 6.5 hours and 8.5 hours, respectively. The main manifestation was testicular pain without additional signs. The results of the laboratory tests did not reflect local advancement. In the 2019 group, Doppler ultrasound showed absent blood flow in the affected testicle in 62% vs. 80% in 2020. The mean time from admission to surgery was virtually identical: 75 minutes in 2019 vs. 76 minutes in 2020. The mean duration of scrotal revision was similar in both groups. There was only one significant difference: the degree of twisting. In 2019, the mean was 360° vs. 540° in 2020. Incidence of orchiectomy also did not significantly vary between the analyzed time periods, with 21% during the pandemic and 35% during the pre-COVID-19 period. *Conclusion.* We did not observe an increase in the number of testicular torsion cases during the COVID-19 pandemic. Most importantly, the rates of orchiectomy did not significantly differ between the patients with testicular torsion presenting during the COVID-19 outbreak.

## 1. Introduction

Acute scrotal pain, with or without scrotal swelling and skin redness, is one of the manifestations of acute scrotum and always requires prompt diagnosis [1]. There are three main causes of acute scrotum in children: testicular torsion, testicular appendage torsion, and epididymo-orchitis [2]. Testicular torsion is one of the most common pediatric emergencies, and it should always be excluded in all patients with acute scrotum. Testicle survival after a torsion event depends primarily on the time of surgical intervention. Early surgery within 6 hours from the onset of symptoms results in a testicular salvage rate of up to 90–97% [3].

In our survey, we wanted to analyze how COVID-19 pandemic lockdown measures influenced the incidence of orchiectomy in boys with testicular torsion. The World Health Organization (WHO) declared the COVID-19 pandemic in March 2020 [4]. In Poland, the first official case of COVID-19 was also reported in March 2020. Despite pandemic restrictions, in our pediatric surgery department, emergency surgery procedures were performed without delay.

The primary purpose of this study was to compare two groups of patients with testicular torsion from two different time periods: before and during the COVID-19 pandemic. More specifically, the cohort comprised boys with testicular torsion treated in the years 2019 and 2020 in our pediatric surgery department. We performed an analysis of their medical histories and focused on clinical symptoms and surgical treatment results to assess the potential impact of the pandemic on treatment outcomes in patients with testicular torsion.

## 2. Materials and Methods

### 2.1. Study Population

This was a single-centre and retrospective cohort study. The inclusion criteria were: pediatric patients aged under 18 years who had undergone emergent surgery due to acute testicular torsion. The exclusion criterion was every other severe or chronic disease. A total of 44 boys aged 1 month–18 years who had undergone emergency scrotal exploration for acute testicular torsion between January 2019 and December 2020 were enrolled into the study. The study protocol was approved by the local Ethics Committee of the Medical University of Bialystok, Poland (APK.002.392.2020).

### 2.2. Data Collection

The patients were divided in two groups. The first group (pre-COVID-19) comprised boys operated on in 2019 and the second one (COVID-19) consisted of children operated on during the COVID-19 pandemic throughout 2020. We compared the two groups in terms of demographic data, local and general symptoms, and treatment outcomes. Laboratory tests and Doppler scrotal ultrasound were performed in all patients. We compared these results and intraoperative findings (degree of torsion, determined by assessing the color of the testicle 5 minutes after detorsion, using an intraoperative scale (ITSC, Intraoperative Testis Color Scale)) [5], methods of surgical intervention, antibiotic therapy, length of operation and hospitalization, and followup. All patients in 2020 were operated after obtaining the result of COVID-19 Antigen Rapid Test. Standard surgical procedures used in our department involved scrotal exploration through a transversal incision, manual testicular detorsion, wrapping the testis with warm saline-soaked gauze, and intraoperative (5 minutes after detorsion) assessment of color of the affected testis on a visual scale (ITSC) [5]: 1—normal/pink, 2—mottled pink/light blue, 3—light blue, 4—dark blue/purple, 5—black, and 6—hemorrhagic/necrotic. We divided the patients into two groups: the first with scores 1–3 and the second with scores 4–6. The next step was orchiectomy or orchiopexy, depending on the viability of the gonad. Testicular fixation was performed by suturing of the tunica albuginea to the dartos layer with 2 or 3 single absorbable 3-0 or 4-0 stitches along the vertical axis and in the lower pole of the testis. In addition, when a testicular appendage was found, it was removed.

### 2.3. Statistical Analysis

Biostatistical processing of the obtained data was performed with the use of GraphPad Prism 9 (GraphPad Software Inc., San Diego, CA, USA). Medians with 25−75th percentiles (interquartile range) were used to summarize the quantitative variables, whereas absolute and relative (percentage) values were used to present qualitative data. For comparison of the differences between studied groups, the nonparametric Mann–Whitney test was used. The Chi-square test was applied for the evaluation of changes in the distribution of qualitative parameters. Relative risk analysis was performed with the use of Fisher's exact test with a 95% confidence interval, calculated using Koopman asymptomatic score. Differences were considered statistically significant with *p*-value below 0.05 and indicated within graphs or tables with exact values or asterisks: ^*∗*^—*p* < 0.05, ^*∗∗*^—*p* < 0.01, ^*∗∗∗*^—*p* < 0.001, and ^*∗∗∗∗*^—*p* < 0.0001.

## 3. Results

Medical charts of 44 children diagnosed and operated on because of testicular torsion in the pediatric surgery and urology department between 2019 and 2020 were analyzed.

The two groups did not differ significantly in terms of age, number of cases, or demographic data (Table 1).

In the year 2019, before the COVID-19 pandemic, 24 boys were operated on because of testicular torsion; their median age was 13.4 years, including three neonates (1-month-old, 6-month-old, and 7-month-old). In the year 2020, during the pandemic, 20 boys were operated on, with a median age of 14.5 years, including one 4-month-old neonate. In both groups, patients lived mainly in urban areas: 58% patients in 2019 and 80% patients in 2020.

In 2019, torsion occurred in the left testis in 71% cases vs. 50% cases in 2020. There were no statistical differences in the duration of symptoms: 8.5 hours (3.25–33.0) in the COVID-19 group vs. 6.5 hours (4.25–22.00) in the pre-COVID-19 one (Table 1).

We analyzed the local and general symptoms of testicular torsion (Table 1). The general symptoms, such as pain location, vomiting, or fever were not statistically different between the COVID-19 period and the pre-COVID-19 year. In both groups, the main manifestation was testicular pain without abdominal pain, fever, or vomiting. In both groups, scrotal edema and erythema predominated among the local symptoms (Table 2).

The results of the laboratory tests did not reflect the status of the gonad. Before the pandemic, the median white blood cell count was 10.33 × 10^9^/L, compared to 11.75 × 10^9^/L during the pandemic. Likewise, the median level of CRP in the first group was 0.66 mg/ml, compared with 0.60 mg/ml in the second (Table 1).

We also analyzed Doppler ultrasound findings (Table 3).

Before the pandemic, in 65% cases testicles were heterogeneous vs. 78% during the pandemic. 45% of the twisted testicles in the first group were described as hypoechoic, 45% as isoechoic, and 10% as hyperechoic vs. 29% as hypoechoic, 50% as isoechoic, and 21% as hyperechoic in the second group. We noticed that in 2019, ultrasound examination showed absence of blood flow in the affected testicle in 62% of cases vs. 80% in 2020. The last parameter that we evaluated using USG was the testicle position. There were four possibilities: transversal, rotated, inguinal, and elevated position. We found no difference between both groups of patients as regards this parameter.

During the pandemic year of 2020, our department did not change the protocols of treatment for testicular torsion, apart from introducing COVID-19 Antigen Rapid Tests before surgery. There were no patients with positive results. The time from admission to surgery was nearly identical: 75 minutes (52.25–98.50) in 2019 vs. 76 minutes (64.50–101.50) in 2020. Furthermore, the mean duration of scrotal revision was also similar: 25 minutes in 2019 vs. 20 minutes in 2020. Likewise, there was no difference in the mean length of hospitalization: 24 hours in both groups. There was a significant difference between the degrees of testicle twisting. In 2019, the mean degree was 360°, while in 2020−540°. Interestingly, a higher degree of testicular rotation did not influence the rate of orchiectomy. Incidence of orchiectomy was also not significantly different between the two time periods: 21% (5/19) in the pre-COVID-19 period and 35% (7/13) during 2020. In both groups, the frequency of testicular appendage torsion was 42% (10/24 and 8/19 cases, respectively). In both groups, the majority of patients fell into the 1–3 categories on the ITSC scale (Table 4).

There was no statistically significant difference in regards to the antibiotic therapy in patients treated in 2019 vs. 2020. However, the variety of protocol treatment was wide (Figure 1).

No perioperative complications were recorded in either of the groups. There were no readmissions during either of the followup periods. Three cases of postoperative testicular atrophy were noted in the pre-COVID-19 group.

We also assessed the relative risk of orchiectomy in the context of selected parameters (Figure 2).

And, it is found that boys without scrotal erythema had more than 7 times lower risk of orchiectomy than patients with this local symptom. The difference was statistically significant. Lack of scrotal edema was associated with a fourfold lower risk of orchiectomy. The risk of testicular loss was 16 times lower when the duration of symptoms was below 12 hours. Similarly, patients with lower scores on the ITCS scale had a 16 times lower risk of orchiectomy. WBC below 10^4^/*μ*l and CRP below 10 mg/ml were also associated with lower risk of orchiectomy (3.5 and 4 times, respectively). In addition, lack of testicular heterogeneity in scrotal ultrasound was associated with a 6 times lower risk of orchiectomy. Similarly, we analyzed the risk of qualification into low [1–3] or high [4–6] ITCS score groups in relation to laboratory parameters and ultrasound findings (Figure 3).

Patients with normal leukocytosis had a 4 times higher chance of a lower score on the ITCS scale. Moreover boys with lower CRP levels had a 2 times greater chance of a lower ITCS score. Patients without testicular heterogeneity in USG had a 4 times higher possibility of being in a low ITSC group. Patients with testicular torsion below 360° had a 2 times higher chance of having a lower ITCS score.

## 4. Discussion

The COVID-19 pandemic posed a challenge not only in terms of providing medical treatment but also in the functioning of the entire healthcare system. Testicular torsion is one of the most time-sensitive paediatric emergencies: surgical intervention during the first few hours from the onset of the symptoms increases the chance of testicular salvage. Similarly to other authors investigating this matter, during the first wave of the outbreak, we did not observe a statistically significant difference in the time from the onset of the symptoms to the admission to the emergency department [6–8]. On the other hand, Pogorelic et al. noted a lengthening of that period to up to 14 hours during the COVID-19 pandemic, which may be the cause of higher rates of orchiectomy in that time in Croatia [9]. Holzman's study [10] also found that the median time from symptom onset to emergency department presentation during COVID-19 was 17.9 hours, and hence, in the COVID-19 group, 42% of patients underwent orchiectomy compared to 29% of the patients with pre-COVID time. Although we did not observe a statistically significant rise in the orchiectomy rate, the median time from the onset of symptoms to admission to hospital has risen from 6.5 hours (2019) to 8.5 hours (2020). Taking into consideration that testicular torsion is one of the most time-sensitive emergencies, 2 hours might result in irreversible changes in the testis which sometimes leads to testicular atrophy and eventually orchiectomy. In the latest population-based study [11] comprising 5,694 patients with testicular torsion, the rate of orchiectomy was 24.78%, with the highest rate in children from 0 to 1 year (45.37%) and males older than 50 years (74.38%). This is similar to another study [12] on 1,713 pediatric patients with testicular torsion and a 28% rate of orchiectomy. Both results are comparable with our findings: we observed a 25% rate of testicular resection in our patients with testicular torsion.

According to Zvizdic et al., the duration of symptoms is the only predictor of testicular salvage [13]. Since the time from the onset of symptoms to access to an emergency department remains under parental control, in our opinion the focus should be placed on providing proper treatment as soon as possible after admission to the hospital, particularly shortening the time to surgery. Our findings reveal no significant differences between the time from admission to surgical treatment or the mean duration of scrotal revision. Therefore, we can conclude that the quality of medical care provided for children in our department during the COVID-19 pandemic was comparable to that during the studied pre-COVID-19 period. According to Gold et al. [14], quality of healthcare is an independent factor determining testicular survival. It seems significant that in our hospital the time from admission to surgery was nearly identical before and during the pandemic period. Moreover, this time was significantly shorter when compared to other analyzes. In a recent study by El-Mezayen et al. the time from admission to surgery was 127–196 minutes [15], while in another by Gold et al. 135 minutes [14]. Although the COVID-19 pandemic has significantly limited access to the healthcare system, and some studies showed delays in admission to EDs and a more severe course of disease, it does not seem to have affected patients with testicular torsion [16, 17]. This may be due to the significantly smaller number of COVID-positive pediatric patients compared to adults [18]. On the other hand, neither patients, nor caregivers, underestimated disturbing symptoms such as acute testicular pain.

According to our survey, the typical patient with testicular torsion is a teenager with acute pain of the left testicle, without other local or general symptoms. Despite the high sensitivity and specificity of Doppler scrotal ultrasound, this investigation does not always provide an accurate diagnosis [19]. Nevertheless, as recommended by our protocol, we performed ultrasound in all patients. Typical findings were heterogeneity of the gonads and abnormal testicle position. Absence of blood flow in the gonads in ultrasound examination was found in 71% cases and did not correlate with the rate of orchiectomy (25%). It needs to be highlighted that surgical exploration must be performed every time when history and symptoms indicate acute testicular torsion, regardless of the result of Doppler scrotal ultrasound. Biochemical blood results did not correlate with the local symptoms. However, normal WBC and CRP levels were more commonly observed in patients with lower ITCS scores. It should be added that there are no clear guidelines on antibiotic prophylaxis. In our center, all patients with testicular torsion received antibiotic treatment, regardless of laboratory results or intraoperative findings.

## 5. Conclusion

New organization of the Polish health care system during the COVID-19 pandemic did not delay proper diagnosis or treatment of testicular torsion in the pediatric population. In conclusion, fear of infection and limited availability of GP care did not affect the rate of surgical orchiectomy after testicular torsion in boys.

## Figures and Tables

**Figure 1:** Antibiotic therapy in patients with testicular torsion.

**Figure 2:** Relative risk of orchiectomy in the context of selected parameters.

**Figure 3:** Risk of qualification into ITCS score groups in relation to laboratory parameters and ultrasound findings. (a) WBC. (b) CRP. (c) Torsion degree. (d) Blood flow presence. (e) Testicular heterogeneity.

**Table 1:** Demographic data and clinical characteristics of the patients. Medians with 25−75th percentiles (interquartile range) were used to summarize the quantitative variables.

Parameters	2019 pre-COVID19	2020 inter-COVID19	*p* value
	(*n* = 24)	(*n* = 20)	
Age (years)	13.4 (3.9; 15.9)	14.5 (13.8; 15.3)	0.3227
Symptoms duration (hours)	6.50 (4.25; 22.00)	8.50 (3.25; 33.00)	0.8744
Area of living (urban/rural)	58%/42% (14/10)	80%/20% (16/4)	0.1244
Testicular torsion side (left/right)	71%/29% (17/7)	50%/50% (10/10)	0.1576
WBC (10^4^ cells/*μ*l)	10.33 (8.40; 11.90)	11.75 (6.85; 13.65)	0.8517
CRP (mg/l)	0.66 (0.30; 7.02)	0.60 (0.30; 2.86)	0.9943
Pain localization (testicular/+abdominal)	79%/21% (19/5)	70%/30% (14/6)	0.4884
Vomiting (yes/no)	21%/79% (5/19)	25%/75% (5/15)	0.7426
Fever (yes/no)	4%/96% (1/23)	0%/100% (0/20)	0.3558
Scrotal edema (yes/no)	38%/62% (9/15)	50%/50% (10/10)	0.4046
Scrotal erythema (yes/no)	21%/79% (5/19)	25%/75% (5/15)	0.7426

**Table 2:** Summary characteristic of all patients with testicular torsion.

Parameters	Testicular torsion patients
	(*n* = 44)
Age (years)	14.1 (12.3; 15.5)
Symptoms duration (hours)	6.50 (4.00; 24.00)
Area of living (urban/rural)	70%/30% (13/13)
Testicular torsion side (left/right)	61%/39% (27/17)
WBC (10^4^ cells/*μ*l)	11.30 (7.65; 13.20)
CRP (mg/l)	0.62 (0.30; 506)
Pain localization (testicular/+abdominal)	75%/25% (33/11)
Vomiting (yes/no)	23%/77% (10/34)
Fever (yes/no)	2%/98% (1/43)
Scrotal edema (yes/no)	43%/57% (19/25)
Scrotal erythema (yes/no)	23%/77% (10/34)
Testicular heterogeneity (yes/no)	69%/31% (20/9)
Testicular echogenicity (hypo-/iso-/hyper-echogenic)	36%/50%/14% (8/11/3)
Blood flow presence (yes/no)	29%/71% (12/29)
Position of the testicle (transversal/rotated/inguinal/elevated)	27%/39%/17/17% (6/9/4/4)
Torsion degree (degree)	360.00 (360.00; 720.00)
ITCS^*∗*^ score (1 − 3/4 − 6)	78%/22% (32/9)
Blood flow restoration (yes/no)	69%/31% (27/12)
Orchiectomy (yes/no)	27%/73% (12/32)
Testicular appendage resection (yes/no)	41%/59% (18/25)
Admission to surgery duration (minutes)	75.00 (60.75; 100.00)
Surgery duration (minutes)	20.00 (20.00; 25.00)
Hospitalization duration (hours)	24.00 (24.00; 48.00)

**Table 3:** Scrotal ultrasound findings.

Parameters	2019 pre-COVID19	2020 inter-COVID19	*p* value
	(*n* = 24)	(*n* = 20)	
Testicular heterogeneity (yes/no)	65%/35% (13/7)	78%/22% (7/2)	0.4914
Testicular echogenicity (hypo-/iso-/hyper-echogenic)	45%/45%/10% (4/4/1)	29%/50%/21% (4/7/2)	0.8030
Blood flow presence (yes/no)	38%/62% (8/13)	20%/80% (4/16)	0.2031
Position of the testicle (transversal/rotated/inguinal/elevated)	29%/36%/21%/14% (4/5/3/2)	22%/45%/11%/22% (2/4/1/2)	0.8673

**Table 4:** Intraoperative findings and treatment of the patients.

Parameters	2019 pre-COVID19	2020 inter-COVID19	*p* value
	(*n* = 24)	(*n* = 20)	
Torsion degree (degree)	360.00^*∗*^ (360.00; 540.00)	540.00^*∗*^ (360.00; 720.00)	**0.0032**
ITCS^*∗*^ score (1 − 3/4 − 6)	87%/13% (20/3)	67%/33% (12/6)	0.1193
Blood flow restoration (yes/no)	77%/23% (17/5)	59%/41% (10/7)	0.2158
Orchiectomy (yes/no)	21%/79% (5/19)	35%/65% (7/13)	0.2934
Testicular appendage resection (yes/no)	42%/58% (10/14)	42%/58% (8/11)	0.9769
Admission to surgery duration (minutes)	75.00 (52.25; 98.50)	76.00 (64.50; 101.50)	0.4231
Surgery duration (minutes)	25.00 (20.00; 29.00)	20.00 (20.00; 25.00)	0.2466
Hospitalization duration (hours)	24.00 (24.00; 48.00)	24.00 (24.00; 24.00)	0.0829

## Data Availability

The data used to support the findings of this study are included within the article.
